The article "Predicting Characteristics Associated with Breast Cancer Survival Using Multiple Machine Learning Approaches" was retracted in 2023. Reasons: unreliable results or conclusions; concerns about the data; concerns about the peer review; concerns about the citations.

# Predicting Characteristics Associated with Breast Cancer Survival Using Multiple Machine Learning Approaches

**DOI:** 10.1155/2022/1249692

**Published:** 2022-04-25

**Authors:** Mohammad Nazmul Haque, Tahia Tazin, Mohammad Monirujjaman Khan, Shahla Faisal, Sobhee Md. Ibraheem, Haneen Algethami, Faris A. Almalki

**Affiliations:** ^1^Department of Electrical and Computer Engineering, North South University, Bashundhara, Dhaka 1229, Bangladesh; ^2^Department of Statistics, Government College University, Faisalabad, Pakistan; ^3^Department of Computer Science, College of Computers and Information Technology, Taif University, P.O. Box 11099, Taif 21944, Saudi Arabia; ^4^Department of Computer Engineering, College of Computers and Information Technology, Taif University, P.O. Box 11099, Taif 21944, Saudi Arabia

## Abstract

Breast cancer is one of the most commonly diagnosed female disorders globally. Numerous studies have been conducted to predict survival markers, although the majority of these analyses were conducted using simple statistical techniques. In lieu of that, this research employed machine learning approaches to develop models for identifying and visualizing relevant prognostic indications of breast cancer survival rates. A comprehensive hospital-based breast cancer dataset was collected from the National Cancer Institute's SEER Program's November 2017 update, which offers population-based cancer statistics. The dataset included female patients diagnosed between 2006 and 2010 with infiltrating duct and lobular carcinoma breast cancer (SEER primary cites recode NOS histology codes 8522/3). The dataset included nine predictor factors and one predictor variable that were linked to the patients' survival status (alive or dead). To identify important prognostic markers associated with breast cancer survival rates, prediction models were constructed using *K*-nearest neighbor (K-NN), decision tree (DT), gradient boosting (GB), random forest (RF), AdaBoost, logistic regression (LR), voting classifier, and support vector machine (SVM). All methods yielded close results in terms of model accuracy and calibration measures, with the lowest achieved from logistic regression (accuracy = 80.57 percent) and the greatest acquired from the random forest (accuracy = 94.64 percent). Notably, the multiple machine learning algorithms utilized in this research achieved high accuracy, suggesting that these approaches might be used as alternative prognostic tools in breast cancer survival studies, especially in the Asian area.

## 1. Introduction

Breast cancer has a high mortality rate. Breast cancer affects more than 1.5 million women worldwide each year, as per the World Health Organization [1]. Breast carcinoma is one of the most well-known kinds of cancer, having been first discovered in Egypt in approximately 1600 BC [2]. Tumors may be used to screen for breast cancer. Tumors are categorized as benign or malignant. To identify malignant neoplasms, physicians must use an active detection strategy. However, even with professionals, cancers are notoriously difficult to detect [3]. As a consequence, an automated technique is required for cancer detection. Numerous studies have tried to predict the survival of carcinoma in humans using machine learning methodologies, and they have also shown that these algorithms are more successful in diagnosing carcinoma [3]. Typically, a physician's knowledge and ability are essential to ensure a patient's detection precision [4]. This capacity, however, is perfected through years of seeing the detrimental effects of various individuals and validating diagnoses. Despite this, there is no guarantee of reliability. Due to developments in processing technology, it is now very simple to collect and maintain large amounts of data, such as specialized databases of electronic patient information [5]. Without the help of a personal computer, it would be difficult to parse these enormous datasets, considerably more so while doing broad information examination. Also, an exact replica of genuine cancer might keep individuals from getting vital therapy. As a result, precisely diagnosing and arranging bosom disease into harmless and threatening subtypes is a significant subject of study. Somewhat recently, AI calculations have been broadly utilized to distinguish bosom diseases and derive different ideas from information designs. AI is well known for its application in disease classification and demonstration. It is a strategy for finding examples of obscure consistency in a wide scope of datasets. It contains an expansive assortment of strategies for uncovering rules, ideal models, and connections inside information groupings, as well as respect to making theories about these linkages that might be used to see recently covered information.  Figure 1 illustrates the primary applications of machine learning in the medical field.

The article "Predicting Characteristics Associated with Breast Cancer Survival Using Multiple Machine Learning Approaches" was retracted in 2023. Reasons: unreliable results or conclusions; concerns about the data; concerns about the peer review; concerns about the citations.

As a consequence, AI's usage in healthcare contexts is quickly growing as a consequence of its predictive and classification capabilities, most notably in clinical analysis to define breast cancer, and it is now extensively utilized in biomedical research.

Breast cancer is still the most prevalent malady among Bangladeshi women. It has developed into a hidden weight, accounting for 69 percent of illness deaths in females [6]. Breast cancer has the greatest prevalence rate (19.3 per 100,000) among Bangladeshi females between the ages of 15 and 44 years [7] when compared to other types of illness. Between 2008 and 2010, cervical cancer was the second most common cancer in this group of women, with a prevalence rate of 12.4 per 100,000. The absence of infection awareness, lack of confidence in clinical decision-making, unethical screening procedures, and early metastatic misuse have all been linked to an increase in the frequency rate [8]. Additionally, patients are prevented from receiving cancer therapy due to a lack of financial resources, the infection's social stigma, and their fear of the treatment. According to findings from research conducted by Bangladesh's National Institute of Cancer Research and Hospital in 2010, breast cancer was responsible for 21% of all deaths among women aged 15 to 49. Bangladesh's National Institute of Cancer and Research Hospital urges that bosom disease become a serious public health concern for the Bangladesh government. According to a study conducted in Bangladesh's Khulna Division in 2007–2008, 87 percent of new cases of bosom illness were classified as stage III+, indicating that malignant development has spread to various body areas. Treatment options were limited and costly, even more so in low-income nations like Bangladesh. The main reason for this could be a lack of public awareness about early cancer screening, which is similar to the case in Bangladesh's rural districts.

Already, specialists have dissected factors influencing bosom malignant growth endurance rates utilizing basic programming projects like Microsoft Excel, SPSS, and STATA [9–11]. These preprogrammed measurable devices are not particularly adaptable when it comes to tracking down new factors or delivering inventive and integrative outlines [12]. Because of the shortcomings of traditional factual examinations, various AI (ML) calculations have been widely used in this domain [13–20]. The choice tree approach is a managed learning method that pictures the results in an effectively interpretable tree structure, which is the basis for breaking down tremendous measures of information [21–24]. Breiman's calculation, a subordinate of DT, is fit for working in both regulated and unaided modes and can deal with both consistent and straight-out information in order and relapse issues [25, 26]. Artificial neural networks have regularly been described as secret elements, demonstrating via preparing on information with known results and tuning loads for further developed expectations in situations with obscure results [27, 28]. Outrageous Boost is a parallelizable outfit of order and relapse trees that produces precise forecasts, is easy to utilize, and has beaten different calculations in different AI challenges [29]. Strategic relapse is based on Gaussian dispersion and is capable of dealing with various types of factors, such as nonstop, discrete, and dichotomous, without making any assumptions about their ordinariness [30, 31]. For regulated grouping, support vector machines are used. They work by defining the best choice limit for isolating main elements into specific groups and then forecasting the class of future perceptions based on this detachment limit [32]. Despite the fact that AI strategies for bosom disease have been created and inspected before, factors like area, way of life, and open information might shift. We confirmed that it is indispensable to foster models for the Bangladeshi setting to learn the factors influencing bosom malignant growth patients' endurance rates. In addition, it is very useful to execute variable choice utilizing AI approaches in the clinical area, where experts have an inclination for old-style factual strategies. The goal of this study is to use conventional AI approaches to develop interpretable prognostic models to uncover the primary characteristics that affect persons with heart disease's survival rates in an Asian climate. The major goal of this study is to demonstrate how machine learning may be used to detect breast cancer features. The study's most significant aspect is that we used a variety of well-known machine learning algorithms to achieve the best results. In our investigation, we used many well-known machine learning algorithms. The RF, DT, K-NN, SVM, voting classifier, GB classifier, AdaBoost classifier, and LR algorithms achieved 94.64 percent, 89.22 percent, 83.87 percent, 84.67 percent, 88.26 percent, 91.78 percent, 89.0 percent, and 80.57 percent accuracy, respectively. The accuracy percentage of the models utilized in this analysis is substantially higher than in earlier investigations, indicating that these models are more reliable. Several model evaluations have demonstrated their resilience, and the strategy may be extrapolated from the study.

The article "Predicting Characteristics Associated with Breast Cancer Survival Using Multiple Machine Learning Approaches" was retracted in 2023. Reasons: unreliable results or conclusions; concerns about the data; concerns about the peer review; concerns about the citations.

According to research, the situation may improve if women can detect and cure breast cancer early. They must do so by accurately forecasting the disease's development from a mild condition to breast cancer. Machine learning technology may aid in the early generation of correct forecasts. There are several machine learning systems, but unfortunately, their predictions are unreliable and inaccurate. They are also concerned about over- and underfitting. As a result, we developed a machine learning model to assist medical technicians in the early detection of cancer sickness. It will confirm and indicate whether or not an individual has breast cancer.

Our study's key contribution, as previously stated, is that we used numerous machine learning models on a publically available dataset. Previously, the majority of research used a large model to predict breast cancer. However, we tested many different machine learning algorithms to predict breast cancer features and compared the results to earlier studies. The remainder of this work is organized as follows.  Section 2 discusses the Method and Experiment Methodology, Section 3 discusses the Result Analysis, and Section 4 discusses the Conclusions.

## 2. Method and Experiment Methodology

This part includes a description of the dataset, a block diagram, a flow diagram, assessment matrices, and information on the techniques and materials utilized.

### 2.1. Dataset

This breast cancer patient database was compiled from the November 2017 update of the National Cancer Institute's SEER Program, which provides population-based cancer statistics [33]. Female patients diagnosed with infiltrating duct and lobular carcinoma breast cancer (SEER primary cites recode NOS histology codes 8522/3) between 2006 and 2010 were included in the study. Patients with uncertain tumor size, patients with investigated regional LNs, patients with positive regional LNs, and patients with less than one month of survival were omitted; hence, 4024 patients were eventually included. The complete number of data in the “status” column of the dataset is shown in Figure 2.

The overall number of missing values in each column of the database is shown in Figure 3. Due to the absence of a missing value, the outcome has been displayed as zero.

### 2.2. Block Diagram of the System

The block diagram of the AI framework is displayed in Figure 4. The components that contribute to the expectation have been identified, and the model's objective value has been established so that it can hypothesize. After that, the dataset was divided into equal portions for preparation and testing. The split was accomplished by random examination, which results in an unequal distribution of preparation and testing time.

Following that, two examinations were conducted, with an 80 percent preparation size and a 20% testing size. Following that, the pieces were scaled using guidelines. To facilitate comprehension, several histogram and scatterplot representations of the preparation split were created. Following that, the framework's preparation begins.

### 2.3. Used Algorithms

Breast cancer is the most commonly detected disease in the medical field, and the incidence of diagnosis is increasing year after year. The SEER Breast Cancer Database was used to assess eight widely used machine learning algorithms for predicting breast cancer recurrence mortality rates.

- Random forest
- Decision tree
- *K*-nearest neighbor
- Logistic regression
- Support vector machine
- Voting classifier
- Gradient boosting classifier
- AdaBoost classifier

The article "Predicting Characteristics Associated with Breast Cancer Survival Using Multiple Machine Learning Approaches" was retracted in 2023. Reasons: unreliable results or conclusions; concerns about the data; concerns about the peer review; concerns about the citations.

#### 2.3.1. Random Forest Flowchart

Random forest is a technique for directed machine learning [34]. It makes a “forest” out of a group of carefully chosen trees that have been largely prepped for the “bagging” technique. The bagging strategy's basic rationale is that mixing many learning models increases the final result. Random forest generates several alternative trees and combines them to get a more precise and dependable representation. It offers the benefit of tackling the arrangement and relapse problems that plague the majority of modern machine learning frameworks. One more striking component of the random forest methodology is that deciding the overall significance of everything in the estimate is so direct. Sklearn offers a remarkable mechanical assembly for assessing the meaning of a component by looking at how much pollution is decreased all throughout the backwoods by the tree communities that utilize it. Following planning, it works out this score for each brand name and changes the discoveries, fully intent on raising the outright importance. The adaptability of the random forest is one of its most charming elements. It can be used to find backslides and gather data, and the importance of good data is clear. Moreover, it is a valuable system since the default hyperparameters it utilizes frequently produce unequivocal assumptions. Because there are not many hyperparameters to begin with, understanding them is essential. Overfitting is a notable issue in AI, yet it seldom happens with the erratic arbitrary timberland classifier. The classifier will not overfit the model if there are sufficient trees in the backwoods. The random forest approach is made up of a progression of decision trees, every one of which is developed by utilizing a bootstrap test from a preparation set. The out-of-pack (OOB) test, which we will talk about later, is 33% of the preparation test that is saved for the end goal of testing. The dataset is then infused with one more case of randomization utilizing highlight packing, expanding its assortment while diminishing the relationship across choice trees. The strategy for anticipating differs as per the situation.

#### 2.3.2. Decision Tree Flowchart

This review utilizes a decision tree classifier. This classifier [35] appears to recursively segment the model space. A prescient worldview acts as a guide between the characteristics of a thing and its qualities [36]. It routinely isolates every potential information result into bits. Each nonleaf hub relates to an element explored, each branch to the result of the trial, and each leaf hub to a judgment or order [36]. The root hub of the tree, which is at the very top, shows the most frequently utilized forecast model. A decision tree's two hubs are the decision hub and the leaf hub. While leaf hubs are the consequence of those decisions and have no additional branches, decision hubs are utilized to settle on those choices and contain a few branches. The results of the tests or decisions are dependent upon the dataset's properties. The decision tree is not difficult to grasp since it repeats the meanings that an individual goes through while settling on a certifiable choice. It could be extremely helpful in settling issues with direction. Think about all the doable answers to an issue. Cleaning information is not needed, however much it is with different strategies.

The article "Predicting Characteristics Associated with Breast Cancer Survival Using Multiple Machine Learning Approaches" was retracted in 2023. Reasons: unreliable results or conclusions; concerns about the data; concerns about the peer review; concerns about the citations.

#### 2.3.3. *K*-Nearest Neighbor

One of the most important AI calculations is the K-NN technique. It is dependent on the learning approach used. The K-NN method admits that the new case and previous cases are interchangeable and assigns the new case to a classification that is similar to the previous classifications. The K-NN calculation keeps up with every single accessible data point and arranges new information accordingly in view of its comparability with recently characterized information. This truly means that using the K-NN approach, new information might be quickly arranged into a distinct classification. The K-NN method can be used for relapsing and grouping, although it is most commonly employed for order difficulties. The K-NN method is nonparametric, which means it makes no assumptions about the data. It is now and then alluded to as a “sluggish student” calculation since it does not gain from the preparation set in a flash, but rather keeps up with and orders the data later. The K-NN approach only saves the information during the preparation stage, and when it gets new information, it sorts it into a class that is generally practically identical to the new information. This review uses the *K*-nearest neighbor classifier, which is one of the most frequently involved order calculations in AI [37]. The *K*-nearest neighbor procedure is a nonparametric technique for characterizing information. This classifier characterizes things as indicated by their proximity to “*k*” nearest neighbors. It is worried about the quick environmental elements of the thing, as opposed to the necessary information conveyance [38].

#### 2.3.4. Logistic Regression

Logistic regression is one of the most frequently utilized AI calculations in the regulated learning approach [39]. It is an estimating approach that utilizes a gathering of free factors to expect an all-out subordinate variable. To estimate the result of a single dependent variable, a logistic regression is used. As a result, the end result should have a clear or discrete character. It very well may be Yes or No, 0 or 1, valid or bogus, etc., but probabilistic qualities somewhere in the range of 0 and 1 are presented rather than exact qualities like 0 and 1. Calculated relapse and direct relapse are moderately comparative in their application. Straight regression is utilized to tackle relapse issues, while logistic regression is utilized to address arrangement hardships. Instead of fitting a relapse line, we utilize logistic regression to fit an “S” molded calculated work that predicts two most extreme qualities (0 or 1). The calculated capacity's bend shows the likelihood of anything, for example, regardless of whether cells are harmful, or regardless of whether a mouse is fat contingent upon its weight. As a result of using both continuous and discrete datasets, calculated relapse is a common AI strategy. It can predict and group new information by using both datasets.

The article "Predicting Characteristics Associated with Breast Cancer Survival Using Multiple Machine Learning Approaches" was retracted in 2023. Reasons: unreliable results or conclusions; concerns about the data; concerns about the peer review; concerns about the citations.

#### 2.3.5. Support Vector Machine

A SVM model is a representation of events as points in space, separated by a substantial gap between examples of distinct classes [40]. Alongside direct arrangement, SVMs can achieve successful nonstraight characterization by verifiably planning their contributions to high-layered include spaces. Support vectors alone; we do not have to stress over different perceptions since the edge is determined utilizing the focuses closest to the hyperplane (support vectors), while calculated relapse characterizes the classifier across all places. Thus, SVM benefits from specific innate speedups.

#### 2.3.6. Voting Classifier

A voting classifier is a kind of AI model that learns from a large number of models and predicts an outcome (class) based on the class that has the best chance of being chosen as the result [41]. It basically totals the consequences of every classifier that is taken care of in the democratic classifier and estimates the result class in view of the class with the biggest democratic greater part. In hard democratic, the extended outcome class is the one with the most votes, i.e., the class that had the highest likelihood of being predicted by all of the classifiers. Accept three classifiers as a starting point for predicting the result class (*A*, *A*, and *B*). As a result of the scenario, the majority of people predicted this. Subsequently, *A* will fill in as the last gauge. The resulting class in delicate democracy is the estimate in view of the normal distribution of the probabilities allotted to that class. Expect that given a contribution to three models, the forecast likelihood for class An is (0.30, 0.47, 0.53) and that for class *B* is (0.30, 0.47, 0.53) (0.20, 0.32, 0.40). Hence, with a normal of 0.4333 for class An and 0.3067 for class *B*, class An is clearly the champ since it had the best normal likelihood of arriving at the midpoint of every classifier.

The article "Predicting Characteristics Associated with Breast Cancer Survival Using Multiple Machine Learning Approaches" was retracted in 2023. Reasons: unreliable results or conclusions; concerns about the data; concerns about the peer review; concerns about the citations.

#### 2.3.7. Gradient Boosting Classifier

Gradient boosting is an AI approach that is regularly utilized for relapse and arrangement applications [42]. It creates an expectation model utilizing an ensemble of frail forecast models, most frequently choice trees. At the point when a choice tree fills in as the frail student, the resultant technique is alluded to as “slope-supported trees.” It regularly beats the arbitrary backwoods. A slope-help tree model is developed in a similar way as other supporting methodologies, but it contrasts in that it permits enhancement of any differentiable misfortune work.

#### 2.3.8. AdaBoost Classifier

Boosting was invented in machine learning to address the issue of whether a collection of weak classifiers might be transformed into a strong classifier [43]. A poor learner or classifier is one that outperforms random guessing. Because it will be made up of a large number of weak classifiers, each of which is better than random, it will be resistant to overfitting. As a poor classifier, a simple threshold on a single feature is usually used. It is positive if the characteristic exceeds the anticipated value; otherwise, it is negative. AdaBoost is an acronym for “adaptive boosting,” a technique for converting weak learners or predictors into strong predictors in order to solve classification issues.

### 2.4. Matrices of Evaluation

Figure 5 depicts the confusion matrix. Machine learning classification models' performance is measured using confusion matrices. To assess the performance of the models created, the confusion matrix was employed.

The confusion matrix shows how accurate our models are at forecasting and how often they predict erroneously. False positives and false negatives were attributed to values that were incorrectly predicted, whilst true positives and true negatives were assigned to values that were correctly predicted. The accuracy, precision-recall trade-off, and AUC of the model were used to assess its performance once all of the estimated parameters were entered into the matrix.

## 3. Result and Data Analysis

### 3.1. Visualization of Feature Selection

Figure 6 depicts the strategy to feature selection. The ability to understand how features are connected to one another is aided by feature selection.

The article "Predicting Characteristics Associated with Breast Cancer Survival Using Multiple Machine Learning Approaches" was retracted in 2023. Reasons: unreliable results or conclusions; concerns about the data; concerns about the peer review; concerns about the citations.

As seen in Figure 6, the primary goal characteristic “status” is positively correlated with all other variables except the surviving months.

### 3.2. Accuracy of the Model

#### 3.2.1. Random Forest

A random forest classifier's classification report is shown in Figure 7.

Among all the other algorithms, it had the highest accuracy (94.64 percent). The random forest model can correctly identify 95% of the characteristics that are associated with breast cancer. A random forest classifier's confusion matrix is shown in Figure 8.

There are 1291 correct guesses and 73 incorrect predictions in this example. This model predicted 642 data as 0 and 649 data as 1. So, this is its correct prediction. However, it also predicted 39 data points to be 0 and 34 data points to be 1. This is an absolutely wrong prediction.

#### 3.2.2. Logistic Regression

Figure 9 demonstrates the classification report of the logistic regression classifier.

Here, logistic regression has achieved 81% accuracy. In this case, this model can correctly identify 81% of the characteristics that are associated with breast cancer.

Figure 10 shows the confusion matrix of the logistic regression classifier.

In this case, there are 1099 correct predictions and 265 erroneous predictions, respectively. This model predicted 572 data as 0 and 527 data as 1. So, this is its correct prediction. However, it also predicted 161 data points to be 0 and 104 data points to be 1. This is an absolutely wrong prediction. In this case, the number of wrong predictions is greater than the random forest. For this reason, the accuracy is less than that of the random forest algorithm.

#### 3.2.3. Support Vector Machine

Figure 11 demonstrates the classification report of the support vector classifier.

Here, support vector machine has achieved 85% accuracy. In this case, this model can correctly identify 85% of the characteristics that are associated with breast cancer.

Figure 12 shows the confusion matrix of the support vector classifier.

There are 1155 correct predictions and 209 false guesses in this case. This model predicted 614 data as 0 and 541 data as 1. So, this is its correct prediction. However, it also predicted 147 data points to be 0 and 62 data points to be 1. This is an absolutely wrong prediction. In this case, the number of wrong predictions is greater than the random forest but lower than the logistic regression. For this reason, the accuracy is less than random forest but greater than logistic regression.

#### 3.2.4. Voting Classifier

Figure 13 shows the classification result of the voting classifier.

The article "Predicting Characteristics Associated with Breast Cancer Survival Using Multiple Machine Learning Approaches" was retracted in 2023. Reasons: unreliable results or conclusions; concerns about the data; concerns about the peer review; concerns about the citations.

The voting classifier model can correctly identify 88% of the characteristics that are associated with breast cancer. For this reason, the accuracy is 88%, which is better than logistic regression and support vector machine. A random forest classifier's confusion matrix is shown in Figure 8.

The voting classifier's confusion matrix is shown in Figure 14.

The number of correct forecasts is 1204 while the number of wrong guesses is 160. This model predicted 610 data as 0 and 594 data as 1. So, this is its correct prediction. However, it also predicted 94 data points to be 0 and 66 data points to be 1. This is an absolutely wrong prediction. In this case, the number of wrong predictions is greater than the random forest but lower than logistic regression and support vector machine. For this reason, the accuracy is less than random forest but greater than logistic regression and support vector machine.

#### 3.2.5. Decision Tree Classifier

The classification result of the decision tree classifier is shown in Figure 15.

The decision tree classifier model can correctly identify 89% of the characteristics that are associated with breast cancer. For this reason, the accuracy is 89% which is better than LR, SVM, and voting classifier.

The decision tree classifier's confusion matrix is shown in Figure 16.

The number of correct and false predictions in this case is 1217 and 147, respectively. This model predicted 595 data as 0 and 622 data as 1. So, this is its correct prediction. However, it also predicted 66 data points to be 0 and 81 data points to be 1. This is an absolutely wrong prediction. In this case, the number of wrong predictions is greater than the random forest but lower than logistic regression and support vector machine. For this reason, the accuracy is less than random forest but greater than logistic regression, support vector machine, and voting classifier.

#### 3.2.6. Decision *K*-Nearest Neighbor Classifier

The *K*-nearest neighbor classifier's classification result is shown in Figure 17.

The K-NN model can correctly identify 84% of the characteristics that are associated with breast cancer. For this reason, the accuracy is 84% which is better than with logistic regression.

The K-NN classifier's confusion matrix is shown in Figure 18.

Here, the number of correct predictions and false predictions is 1144 and 220, respectively. This model predicted 584 data as 0 and 560 data as 1. So, this is its correct prediction. However, it also predicted 128 data points to be 0 and 92 data points to be 1. This is an absolutely wrong prediction. In this case, the number of wrong predictions is greater than the random forest but lower than logistic regression. For this reason, the accuracy is less than random forest but greater than the logistic regression.

The article "Predicting Characteristics Associated with Breast Cancer Survival Using Multiple Machine Learning Approaches" was retracted in 2023. Reasons: unreliable results or conclusions; concerns about the data; concerns about the peer review; concerns about the citations.

#### 3.2.7. Gradient Boosting Classifier

Figure 19 shows the classification result of the GB classifier.

The GB model can correctly identify 92% of the characteristics that are associated with breast cancer. As a result, the accuracy is 92 percent, which is higher than the accuracy of other techniques such as LR, SVM, voting classifier, and K-NN.

Figure 20 depicts the gradient boosting classifier's confusion matrix.

Here, the number of correct predictions and false predictions is 1252 and 112, respectively. This model predicted 635 data as 0 and 617 data as 1. So, this is its correct prediction. However, it also predicted 71 data points to be 0 and 41 data points to be 1. This is an absolutely wrong prediction. In this case, the number of wrong predictions is greater than the random forest. But it achieved the second-highest accuracy among all other algorithms.

#### 3.2.8. AdaBoost Classifier

The classification result of the AdaBoost classifier is shown in Figure 21.

The AdaBoost model can correctly identify 89% of the characteristics that are associated with breast cancer. For this reason, the accuracy is 89% which is equal to the decision tree classifier's result.

The confusion matrix of the AdaBoost classifier is shown in Figure 22.

Here, the number of correct predictions and false predictions is 1214 and 150, respectively. This model predicted 621 data as 0 and 593 data as 1. So, this is its correct prediction. However, it also predicted 95 data points to be 0 and 55 data points to be 1. This is an absolutely wrong prediction. In this case, the number of wrong predictions is greater than the random forest.

### 3.3. Model Comparison

The models in Table 1 are compared to those in prior research articles. The table demonstrates unequivocally that random forest is the greatest model among the framework's several models. It has a higher *F*1 score, is more precise, has a better evaluation, and has a larger zone under the bend.

According to Table 1, all of the methods have a good level of accuracy. The random forest approach, on the other hand, is a better option because it is more accurate. In this study, the RF method was 94% accurate. The voting classifier was only 87% accurate in [20]. Using the decision tree method, this article got 89.22 percent of the time right, while the authors of [26] got 73.2 percent of the time right.

## 4. Conclusion

This research used machine learning methods to analyze predictive markers for breast cancer survival. When compared to other algorithms, the random forest approach produced somewhat higher accuracy when evaluating models. In this research, RF, DT, K-NN, SVM, voting classifier, GB classifier, AdaBoost classifier, and LR algorithms achieved 94.64 percent, 89.22 percent, 83.87 percent, 84.67 percent, 88.26 percent, 91.78 percent, 89.0 percent, and 80.57 percent accuracy, respectively. Nonetheless, the accuracy of all the algorithms looked to be near. In this regard, this research established the model's performance and significant factors affecting breast cancer patients' survival rates, which may be used in clinical practice, especially in the Asian scenario. The accuracy % of the models used in this study is significantly greater than in previous research, implying that the models used in this study are more accurate. The random forest technique beats other approaches when cross-validation measures are used to predict breast cancer. The framework models could be improved in the future by adding a larger dataset and machine learning models like majority voting and bagging. This increases the framework's reliability and enhances its presentation. By simply submitting MRI data, the machine learning framework may assist the general community in determining the risk of cancer in adult patients. Ideally, it will aid patients in obtaining early cancer treatment and reclaiming their lives.

The article "Predicting Characteristics Associated with Breast Cancer Survival Using Multiple Machine Learning Approaches" was retracted in 2023. Reasons: unreliable results or conclusions; concerns about the data; concerns about the peer review; concerns about the citations.

## Figures and Tables

**Figure 1:** Application of machine learning in the medical field.

**Figure 2:** Total number of data in the “status” column after preprocessing.

**Figure 3:** Outcome of missing data.

**Figure 4:** System block diagram.

**Figure 5:** Block diagram of confusion matrix.

**Figure 6:** Visualization of feature selection.

**Figure 7:** Random forest classifier classification report.

**Figure 8:** Confusion matrix of random forest classifier.

**Figure 9:** Classification report of logistic regression classifier.

**Figure 10:** Confusion matrix of logistic regression classifier.

**Figure 11:** Support vector classifier classification report.

**Figure 12:** Confusion matrix of support vector classifier.

**Figure 13:** Voting classifier's classification report.

**Figure 14:** Confusion matrix of voting classifier.

**Figure 15:** Decision tree classifier classification report.

**Figure 16:** Confusion matrix of decision tree classifier.

**Figure 17:** Classification report of K-NN classifier.

**Figure 18:** Confusion matrix of *K*-nearest neighbor classifier.

**Figure 19:** Classification report of gradient boosting classifier.

**Figure 20:** Gradient boosting classifier confusion matrix.

**Figure 21:** Classification result of AdaBoost classifier.

The article "Predicting Characteristics Associated with Breast Cancer Survival Using Multiple Machine Learning Approaches" was retracted in 2023. Reasons: unreliable results or conclusions; concerns about the data; concerns about the peer review; concerns about the citations.

**Figure 22:** Confusion matrix of AdaBoost classifier.

**Table 1:** Model comparison.

This paper (model name)	Accuracy (%)	Reference paper (model name)	Accuracy (%)
Random forest	94.64	Ref. [20] voting classifier	87.13
Decision tree	89.22	Ref. [26] decision tree	73.2
*K*-nearest neighbor	83.87	Ref. [29] *K*-nearest neighbor	85.0
Logistic regression	80.57	Ref. [31] logistic regression	89.2

## Data Availability

The data used to support the findings of this study are freely available at https://http://ieee-dataport.org/open-access/seer-breast-cancer-data.
